The article "A review of the mechanisms of abnormal ceramide metabolism in type 2 diabetes mellitus, Alzheimer’s disease, and their co-morbidities" was published in 2024. Journal: Front Pharmacol.

# A review of the mechanisms of abnormal ceramide metabolism in type 2 diabetes mellitus, Alzheimer’s disease, and their co-morbidities

**DOI:** 10.3389/fphar.2024.1348410

**Published:** 2024-02-06

**Authors:** Yun Pan, Jieying Li, Panjie Lin, Lihua Wan, Yiqian Qu, Lingyong Cao, Lei Wang

**Affiliations:** School of Basic Medical Sciences, Zhejiang Chinese Medical University, Hangzhou, Zhejiang, China

**Keywords:** ceramide, Alzheimer's disease, type 2 diabetes mellitus, insulin signaling, comorbidity, inflammation

## Abstract

The global prevalence of type 2 diabetes mellitus (T2DM) and Alzheimer’s disease (AD) is rapidly increasing, revealing a strong association between these two diseases. Currently, there are no curative medication available for the comorbidity of T2DM and AD. Ceramides are structural components of cell membrane lipids and act as signal molecules regulating cell homeostasis. Their synthesis and degradation play crucial roles in maintaining metabolic balance *in vivo*, serving as important mediators in the development of neurodegenerative and metabolic disorders. Abnormal ceramide metabolism disrupts intracellular signaling, induces oxidative stress, activates inflammatory factors, and impacts glucose and lipid homeostasis in metabolism-related tissues like the liver, skeletal muscle, and adipose tissue, driving the occurrence and progression of T2DM. The connection between changes in ceramide levels in the brain, amyloid β accumulation, and tau hyper-phosphorylation is evident. Additionally, ceramide regulates cell survival and apoptosis through related signaling pathways, actively participating in the occurrence and progression of AD. Regulatory enzymes, their metabolites, and signaling pathways impact core pathological molecular mechanisms shared by T2DM and AD, such as insulin resistance and inflammatory response. Consequently, regulating ceramide metabolism may become a potential therapeutic target and intervention for the comorbidity of T2DM and AD. The paper comprehensively summarizes and discusses the role of ceramide and its metabolites in the pathogenesis of T2DM and AD, as well as the latest progress in the treatment of T2DM with AD.

## 1 Introduction

Lipids constitute a crucial and remarkably diverse class of molecules, playing pivotal roles in bioenergetics including cyto-architecture, extracellular signaling, and energy storage. Sphingolipids account for 10%–20% of total cellular lipids, with ceramides being the central molecule in overall sphingolipid metabolism (Abou-Ghali and Stiban, 2015). Ceramide, a key precursor of most complex sphingolipids, is synthesized primarily through the *de novo* synthesis pathway, sphingomyelin metabolism pathway, and salvage pathway, utilizing sphingosine as its structural foundation (Zietzer et al., 2022). The cellular ceramide level depends on the balance between production and degradation rates. An imbalance in ceramide metabolism can lead to various chronic diseases, including metabolic, cardiovascular, autoimmune and neurodegenerative diseases (Pilátová et al., 2023). Recent studies have shown that ceramides and their metabolites play key roles in metabolic diseases such as AD, T2DM and neurodegenerative diseases, such as insulin and IGF-1 (Mei et al., 2023). With the aging population, the global prevalence of T2DM and AD is markedly increasing. Notably, the Rotterdam study in the 1990s revealed a twofold increase in the risk of dementia and AD among T2DM patients (Ott et al., 1999). Extensive epidemiological data suggest a strong association between T2DM and an elevated incidence of AD, particularly in patients with multiple clinical comorbidities. Moreover, many similarities in the pathogenesis of T2DM and AD have been observed (Stanciu et al., 2020; Ren et al., 2023). This paper systematically explores the common pathological mechanism of T2DM and AD, identifying ceramide as a central factor in the pathogenesis. The modulation of ceramide metabolism emerges as a potential avenue for treating these comorbidities. In conclusion, ceramide and its metabolites present promising therapeutic targets for addressing T2DM.and AD.

The article "A review of the mechanisms of abnormal ceramide metabolism in type 2 diabetes mellitus, Alzheimer’s disease, and their co-morbidities" was published in 2024. Journal: Front Pharmacol.

## 2 Basic overview of ceramide

Sphingolipids constitute a class of intricate compounds characterized by sphingosine as the skeleton structure, linked to a long chain of fatty acids at one terminus and a polar alcohol structure at the other. These compounds serve as crucial structural elements in biofilms, extensively present in the membrane structures of eukaryotic cells, including cellular and organelle membranes. They play an important role in maintaining biofilm barrier function and fluidity (Spiegel and Merrill, 1996). Beyond their structural significance, sphingolipids also function as essential signaling molecules integral to various biological processes. They actively participate in the regulation of numerous cellular signal transduction processes under both normal and pathophysiological conditions (Merrill et al., 1997; Quinville et al., 2021).

One of the most crucial and basic forms of sphingolipids is ceramide. Ceramide is a core molecule of the overall sphingolipid metabolism and serves as a vital precursor for the majority of complex sphingolipids. Its regulatory capabilities extend to essential cellular processes such as growth, differentiation, senescence, and apoptosis. Ceramide functions as a second messenger within cells, actively participating in diverse signal transduction pathways, immune response regulation, and inflammatory responses (Hammerschmidt and Brüning, 2022). Recognized as a pivotal bioactive lipid, ceramide plays a multifaceted role in cellular dynamics and signaling.

The article "A review of the mechanisms of abnormal ceramide metabolism in type 2 diabetes mellitus, Alzheimer’s disease, and their co-morbidities" was published in 2024. Journal: Front Pharmacol.

As the central point of sphingolipid metabolism, the synthesis and metabolism of ceramide in the body are rigorously regulated. Three primary synthesis pathways govern this process, including *de novo* synthesis pathway, sphingomyelin metabolism pathway and remediation pathway (Clarke et al., 2020). *De novo* synthesis takes place on the cytosolic surface of the endoplasmic reticulum, where serine palmitoyl transferase (SPT) catalyzes the condensation of serine and palmitoyl Coenzyme A, forming 3-keto sphingosine. This compound is then converted to dihydrosphingosine by 3-keto sphingonine reductase. Subsequently CerS1 to CerS6 of Cer synthase (CerS) catalyze the formation of ceramide containing diverse chain-length fatty acids, ensuring specific tissue distribution and physiological function (Bandet et al., 2019). The *de novo* synthesis pathway stands as the principal source of cellular ceramide, accessible to all eukaryotic cells. This pathway has been demonstrated to be the primary synthesis route activated under conditions of obesity and lipid excess (Bandet et al., 2019). Sphingomyelin and ceramide interaction is facilitated by sphingomyelinase and sphingomyelin synthase. Sphingingomyelinase hydrolyzes sphingomyelin or glycosidase hydrolyzes glycosphingolipids, generating ceramide in lysosomes (Maceyka and Spiegel, 2014). Stimulation of cells by factors such as oxidative stress, radiation, or tumor necrosis factor prompts the sphingolipid metabolism pathway to rapidly produce numerous ceramides. Ceramidase catalyzes the hydrolysis of ceramide, producing sphingosine. This sphingosine, recycled through the salvage pathway, contributes to ceramide production, with at least half of sphingosine being reused. The salvage pathway plays a pivotal role in maintaining ceramide homeostasis (Kitatani et al., 2008). In the pathogenesis of T2DM and AD, all three ceramide synthesis pathways are affected. An increase in ceramide levels is associated with disease promotion (Figure 1).

**FIGURE 1:** Schematic of ceramide metabolism.

## 3 Abnormal ceramide metabolism leads to the pathogenesis of T2DM

T2DM is a chronic metabolic disease characterized by hyperglycemia. In 2021, 537 million people were diagnosed with diabetes, and this number is projected to increase to 643 million by 2030 and 783 million by 2045(IDF Diabetes Atlas 10th Edition, n. d.). T2DM, accounting for 90%–95% of cases, is also known as non-insulin-dependent diabetes mellitus. The pathological mechanism of T2DM primarily involves insulin resistance and impaired islet β -cell function. As early as the early 1990s, studies identified the accumulation of specific sphingolipids, particularly ceramide, in the liver and muscle of obese and diabetic rats (Turinsky et al., 1990). Recent clinical studies have further demonstrated a substantial increase in both plasma and urinary ceramide levels in T2DM patients, suggesting ceramide could be used as a potential clinical evaluation index for T2DM (Chew et al., 2019; Nehus et al., 2024). Additionally, the ceramide content in the serum of T2DM patients exhibited a positive correlation with blood glucose value, body weight, and total triglycerides (Wang J. et al., 2023). Ceramide is known to stimulate fatty acids uptake. And its accumulation within cells contribute to significant changes in membrane structure and alterations in cell signaling, thereby affecting the onset and progression of T2DM(Bartke and Hannun, 2009). The influence of ceramide on T2DM manifests through three main aspects: affecting insulin resistance, triggering endoplasmic reticulum (ER) stress, and inducing mitochondrial dysfunction (Li, 2022).

The article "A review of the mechanisms of abnormal ceramide metabolism in type 2 diabetes mellitus, Alzheimer’s disease, and their co-morbidities" was published in 2024. Journal: Front Pharmacol.

### 3.1 Insulin resistance

Insulin, primarily secreted by islet β-cells, plays a pivotal role in regulating glucose metabolism in peripheral tissues. Defective islet β-cell function, leading to reduced insulin secretion, is a prominent pathophysiological characteristic of T2DM(Yang et al., 2023). Hepatic insulin resistance is a major factor in the pathogenesis of T2DM. Ceramides act as key mediators that connect lipid-induced inflammatory pathways to insulin resistance and the development of T2DM(El-Amouri et al., 2023). Notably, the reduction of hepatic ceramide has demonstrated the capacity to ameliorate metabolic disorders, including hepatic insulin resistance (Bzdęga et al., 2023; de Hart et al., 2023). Exposure of muscle cells to saturated fatty acids (e.g., palmitate) attenuates the insulin activation associated with glycogen synthesis and glucose transport, while elevating the intracellular ceramide content (Powell et al., 2004). A study found that a significant positive correlation between intrahepatic ceramide accumulation and blood glucose levels in obese diabetic patients, highlighting ceramide’s potential role in inducing hepatic insulin resistance (Razak Hady et al., 2019). Meanwhile, obesity and insulin resistance coincides with heightened lipid accumulation, including sphingolipids like ceramides (Ciaraldi et al., 2016). Notably, four plasma ceramides (C16:0, C18:0, C20:0, C22:0) were negatively associated with insulin sensitivity and displayed variations over time. Among them, C18:0 is specifically associated with the risk of developing T2DM, and may serve as a potential marker for assessing the risk of T2DM development (Bae et al., 2023).

The article "A review of the mechanisms of abnormal ceramide metabolism in type 2 diabetes mellitus, Alzheimer’s disease, and their co-morbidities" was published in 2024. Journal: Front Pharmacol.

Ceramide disrupts insulin signaling pathways through three major ways. Firstly, ceramide production is triggered by the upstream activation of the pro-inflammatory toll-like receptor 4 (TLR4). TLR4 activation by saturated fatty acids is a pathway of innate immunity leading to increased inflammation associated with obesity (Ritter et al., 2015). The mechanism through which TLR4 induces insulin resistance involves the increased transcription of genes associated with ceramide synthesis via IKKβ and NF- κB. These genes, in turn, result in elevated ceramide levels, inhibiting Akt, a crucial component in insulin signaling (Holland et al., 2011). A study using TLR4 function in hematopoietic cell TLR4 mutant virus knockout mice observed increased insulin sensitivity and reduced inflammation. Thus, TLR4 emerges not only as a critical receptor in the inflammatory pathway but also plays a pivotal role in the development of insulin resistance (Saberi et al., 2009).

Secondly, ceramide exerts its influence by suppressing the Akt signaling pathway. Ceramide regulates glucose uptake, lipolysis, gluconeogenesis, and antiglycogen synthesis, leading to insulin resistance by inhibiting Akt-mediated GLUT 4 translocation (Hage Hassan et al., 2016; Samuel and Shulman, 2016). Specifically, ceramide activates protein phosphatase 2 (PP2A) through the protein kinase C (PKC) isoform, PKC ζ, thereby dephosphorylating Akt. Thus, this inhibits Akt’s transport to the plasma membrane, disrupts the Akt/PKB pathway, reduced GLUT 4 expression levels, and perturbs the glucose transporter pathway, leading to insulin resistance (Mandal et al., 2021). In hepatocytes, glucagon enhances PP2A activation, with ceramide further supporting PP2A activation and dephosphorylation of transcriptional coactivator 2 (CRTC 2). CRTC 2 translocates into the nucleus and binds to CREB to form a transcriptional complex and induce its activity, consequently causing gluconeogenic gene transcription and diabetes (Wang J. et al., 2023). The application of PP2A inhibitors proves effective in mitigating ceramide-induced inhibition on Akt/PKB, restoring insulin signaling (Chavez and Summers, 2003; Stratford et al., 2004), and effectively facilitating CRTC 2 phosphorylation regulated by cAMP reactive element binding protein (CREB) in hepatocytes. This, in turn, inhibits CRTC 2 in the cytosol, curbing hepatic gluconeogenesis (Wang J. et al., 2023). In addition, ceramide activates PKC and the activated PKC phosphorylates Thr 34 on Akt, resulting in the recruitment of Akt to the cytoplasmic membrane, impairing insulin signaling (Maceyka et al., 2012). According to the salvage pathway of ceramide, ceramidase facilitates the production of sphingosine, which is then phosphorylated to sphingosine-1-phosphate (S1P) by sphingosine kinase (Kitatani et al., 2008). S1P has been shown to ameliorate insulin resistance and enhance glucose uptake by activating the Akt signaling pathway.

The article "A review of the mechanisms of abnormal ceramide metabolism in type 2 diabetes mellitus, Alzheimer’s disease, and their co-morbidities" was published in 2024. Journal: Front Pharmacol.

The third scenario involves ceramide inducing apoptosis in islet β-cells, crucial producers of insulin with a pivotal role in the pathophysiology of diabetes mellitus. Ceramides have been recognized as important mediators of fatty acid-induced cytotoxicity in β cells. Ceramide increases the release of cytochrome c, triggering the apoptotic pathway in islet β cells (Yaribeygi et al., 2020). In islet cells, ceramide promotes insulin resistance and apoptosis of β cells through the ERK1/2 signaling pathway. In a diabetic rat model, the precursor sphingolipid palmitate of ceramide amplifies β-cell apoptosis through ceramide activation. Ceramide is associated with increased mitochondrial damage, oxidative stress, and ion channel inhibition, all of which are associated with β-cell apoptosis (Guo et al., 2010). In conclusion, ceramide actively contributes to the development of insulin resistance, and targeting ceramide synthesis inhibition may be a potential therapeutic target for T2DM.

### 3.2 ER stress

The ER is an organelle that plays a key role in protein synthesis and folding as well as lipid synthesis. Alterations in ER membrane components can modulate the ER protein folding environment, thereby inducing ER stress. T2DM, characterized by elevated levels of glucose and free fatty acids, leads to β-cell dysfunction or even death in a prolonged high-fat-high-glucose environment (Swisa et al., 2017). Studies have shown that ceramide-induced ER stress plays an important role in the mechanism of glucolipotoxicity-induced β-cell dysfunction (Liu et al., 2023). The *de novo* ceramide synthesis initiates in the cytoplasmic leaflet of the ER membrane, and ceramide plays a key role in regulating membrane thickness and stability (Venkatesan et al., 2023). Ceramide accumulation induces ER stress by increasing protein misfolding and aggregation, and perturbs calcium signaling in the ER (Boslem et al., 2013; Chen et al., 2023). In INS-1 cells, Ceramide promotes ER stress and affects the synthesis and release of insulin (Lei et al., 2008). Glucolipotoxicity inhibits the PI3K/Akt pathway, impairing vesicular transport of ceramide from the ER to the Golgi (Kim et al., 2005; Martinez et al., 2008). In islet β-cells, glucolipotoxicity reduces the synthesis rate of the ceramide transporter CERT, highly phosphorylateing CERT, preventing accurate Golgi localization. Under T2DM glucolipotoxicity, the total amount of CERT decreased, and CERT activity is very low, hindering ceramide transport from the ER to the Golgi and reducing ceramide utilization rates, promoting ceramide accumulation in the ER (Gjoni et al., 2014).

The article "A review of the mechanisms of abnormal ceramide metabolism in type 2 diabetes mellitus, Alzheimer’s disease, and their co-morbidities" was published in 2024. Journal: Front Pharmacol.

Loss of fat storage-inducing transmembrane protein 2 (FIT2) and lipid droplets (LDs) in β-cells lowers β-cell ATP levels, increases intracellular ceramide C16: 0 accumulation, stimulates ER stress, diminishes calcium signaling, inhibits vesicle exocytosis, downregulates β-cell transcription factors, upregulates unfolded protein response genes, and reduces insulin secretion, exacerbating diet-induced T2DM. Inhibiting CerS ameliorates enhanced ER stress and improves insulin secretion (Zheng et al., 2022). Reducing serum ceramide concentration can regulate hepatic ER stress-related proteins, including PERK, ATF6α, CHOP and GRP78BIP, thereby mitigating ER stress and insulin resistance induced by a high-fat diet. This protective measure safeguards islet β-cells, improves glucose and lipid metabolism in T2DM(Xie et al., 2017; Yilmaz, 2017).

### 3.3 Mitochondrial dysfunction

Mitochondria, abundant organelles in most cells, consist of specialized component with multiple physiological functions: the outer mitochondrial membrane, the interstitial mitochondrial membrane, the inner mitochondrial membrane, and the mitochondrial matrix. T2DM is closely related to various forms of mitochondrial dysfunction, including abnormal energy metabolism, imbalance in calcium signal transduction, increased production of reactive oxygen species (ROS), impaired mitochondrial dynamics, and mitophagy (Dadsena et al., 2019; Diaz-Vegas et al., 2023). These dysfunctions can exacerbate insulin resistance and induce cell apoptosis by impacting energy metabolism and promoting oxidative stress. Mitochondria play a vital role in ATP generation through β-oxidation, the citric acid cycle, and oxidative phosphorylation (OXPHOS). ATP synthesis, a hallmark of mitochondrial function, actively participates in various metabolic reactions (Warren et al., 2020). Mitochondrial dysfunction significantly disrupts the normal metabolic process of fatty acids and proteins, and lead to further aggravation of insulin resistance. Ceramide plays an important role in mitochondria function and morphology. Ceramide, crucial in mitochondrial function and morphology, is closely associated with the site of *de novo* ceramide synthesis in the ER. The physical and functional interaction between mitochondria and ER occurs through mitochondrial-associated membranes While ceramides are essential components of mitochondrial membranes and are required for normal mitochondrial function, excessive mitochondrial ceramide content has been shown to increase oxidative stress by producing reactive oxygen species and altering mitochondrial outer membrane permeability. This leads to the release of cytochrome c, inducing mitochondrial dysfunction (Dadsena et al., 2019). For example, elevated ceramide levels in the mitochondria of skeletal muscle cells cause coenzyme Q depletion and loss of the mitochondrial respiratory chain components, resulting in mitochondrial dysfunction and insulin resistance (Diaz-Vegas et al., 2023). Ceramides can directly transfer to mitochondria through the mitochondria-associated membrane (MAM). Long-chain fatty acids are precursors in the *de novo* synthesis of ceramides and play a central role in lipotoxic mitochondrial dysfunction (Chaurasia and Summers, 2021). High glucose levels can promote the synthesis of CerS6 through TLR4/IKKβ pathway, producing ceramide C16:0 (Li et al., 2023). This ceramide stimulates mitochondrial fission through the recruitment of dynamin-related protein 1 (DRP1), increasing mitochondrial oxidative stress and leading to insulin resistance (Hammerschmidt et al., 2019). In high-fat fed mouse models, increased ceramide in liver mitochondria and decreased mitochondrial turnover rate result in mitochondrial metabolic disorders (Mucinski et al., 2023). Ceramide accumulation inhibits hormone-sensitive triglyceride lipase (HSL), leading to excessive lipid storage and impaired mitochondrial function (Gaggini et al., 2022). In diabetes, ceramide glycosylation forms lactose ceramide (LacCer), resulting in mitochondrial dysfunction and reduced energy production. Increased LacCer levels activate superoxide production and multiple signaling pathways, leading to increased inflammation, apoptosis, and oxidative stress (Balram et al., 2022). In T2DM rats, inhibition of ceramide in the ileum increased the activity of hepatic mitochondrial marker Citrate synthase, subsequently decreasing hepatic mitochondrial acetyl CoA level and hepatic Phosphatidylcholine activity. This inhibition proves effective in limiting gluconeogenesis, enhancing glucose metabolism, and ameliorating T2DM symptoms (Zhou et al., 2021). In isolated submuscular and interfibrous mitochondria from streptozotocin (STZ)-treated mouse hearts, many ceramide species do not exhibit an increase. However, during diabetic nephropathy, ceramide accumulation impedes mitophagy, restricting the removal of damaged mitochondria (Wang X. et al., 2023).

The article "A review of the mechanisms of abnormal ceramide metabolism in type 2 diabetes mellitus, Alzheimer’s disease, and their co-morbidities" was published in 2024. Journal: Front Pharmacol.

Therefore, ceramide significantly affects the morphology and function of mitochondria, thereby influencing the body’s normal metabolic processes and contributing to the onset and progression of T2DM (Figure 2).

**FIGURE 2:** The pathogenesis of T2DM caused by ceramides.

## 4 The pathogenesis of ceramide and AD

AD is a neurodegenerative disease characterized by a subtle onset and gradual, progressive deterioration. It is one of the most common types of dementia among the elderly, accounting for 50%–70% of senile dementia cases (Lee et al., 2021). The characteristic pathological changes of AD mainly include Aβ accumulation hypothesis, tau protein hyperphosphorylation hypothesis, APOE metabolic reprogramming hypothesis, α-Syn hypothesis, etc .,(Wang et al., 2024). The deposited Aβ aggregates play a dual role in AD development, acting both as insoluble Aβ in conjunction with ganglioside GM1 and contributing to the formation of extracellular neuroinflammatory Senile Plaques (SP) and Neurofibrillary Tangles (NFTs) formed by tau protein hyperphosphorylation. This, in turn, results in cortical shrinkage, neuronal loss, and synaptic dysfunction, further advancing AD progression (Akyol et al., 2023). The pathological focus of AD centers on the central nervous system (CNS), rich in lipids crucial for membrane fluidity control, cell signaling, and second messenger generation (Alaamery et al., 2021). Over the past few decades, research has identified abnormal ceramide and its metabolites related to the pathophysiology of AD, influencing Aβ accumulation and tau protein hyperphosphorylation, consequently impacting the severity of AD. In the early stages of AD, there is an observed deficiency in multiple glucosides and elevated Cer in the lesion area (Han et al., 2002). Lipidomics studies have revealed a threefold increase in ceramide levels in the brains of AD patients compared to healthy controls (Chowdhury et al., 2022; Reveglia et al., 2023). Elevated plasma ceramide and sphingomyelin levels have also been found in AD patients and have been proposed as diagnostic markers for these diseases (Olsen and Færgeman, 2017). Moreover, ceramide is implicated in causing mitochondrial dysfunction, brain insulin resistance, and promoting neuroinflammation, collectively contributing to the onset and progression of AD (Brodowicz et al., 2018).

### 4.1 Aβ accumulate

Aβ is produced by the proteolysis of Amyloid precursor protein (APP) by β-secretase and γ-secretase. Normally, Aβ is cleared by homeostatic clearance mechanisms and does not accumulate in the brain. However, imbalance between Aβ production and clearance can lead to amyloid plaque formation (Shimada et al., 2017). Neurons, the fundamental structural and functional units of CNS, rely on mitochondria for energy ATP production and calcium homeostasis (Johnson et al., 2023). The abnormal aggregation of Aβ disrupts neuronal structure and function, causing substantial damage to neurons in the brains of AD patients, a primary factor in the pathogenesis of AD. Studies have shown that ceramide is closely related to the formation and aggregation of Aβ. In the brain, ceramides can dysregulate mitochondria, aggravate ER stress, produce excessive reactive oxygen species, and disrupt protein homeostasis, leading to abnormal Aβ accumulation and neuronal apoptosis (Kogot-Levin and Saada, 2014). The expression level of ceramide also affects the content of Aβ, subsequently impacting the progression of AD. γ-secretase activity and Aβ secretion are positively regulated by sphingolipid hydrolases (Yin, 2023). Ceramide directly promotes Aβ production by increasing the stability of β-secretase. Simultaneously, ceramide contributes to a positive feedback loop, inducing oxidative stress response, activating Sphingomyelinase (SMase), and catalyzing the breakdown of sphingomyelin to generate ceramide. This creates a vicious cycle, increasing Aβ deposition, triggering neuronal cell death and neuroinflammation, and aggravating the condition of AD (Jazvinšćak Jembrek et al., 2015). In the female APP NL-F mouse model, increased ceramide C20:0 and total APP/Aβ led to elevated Aβ amyloid load. Inhibition of nSMase2 by GW4869 resulted in a reduction of Aβ plaques in female APP NL-F mice (Mowry et al., 2023). Ceramide transporters (CERTs), particularly the long isomer CERTL, play a crucial role in regulating the balance between ceramides and sphingomyelin. CERTL inhibits Aβ aggregation and reduces Aβ neurotoxicity by binding to APP. In the familial AD transgenic mouse model 5x FAD mouse, overexpression of CERTL reduced Aβ production by decreasing ceramide levels and increasing sphingomyelin content (Crivelli et al., 2021).

The article "A review of the mechanisms of abnormal ceramide metabolism in type 2 diabetes mellitus, Alzheimer’s disease, and their co-morbidities" was published in 2024. Journal: Front Pharmacol.

According to the amyloid hypothesis, the current pathophysiological explanation for AD, elevated Aβ levels in the brain initiate a pathogenic cascade. Elevated Aβ levels ultimately lead to neuronal damage and death, culminating in progressive cognitive deficits. Therefore, an excessive of ceramide can promote the production of Aβ in various forms, and impede the clearance of Aβ in the brain. This dual effect accelerates neuronal damage, contributing to the onset and progression of AD.

### 4.2 Hyperphosphorylation of the tau protein

Tau is abundantly distributed in neurons and plays a role in maintaining the stability of cytoskeletal microtubules and axonal transport (Poorkaj et al., 2001). Neurofibrillary tangles (NFTS) observed in the brains of AD patients are a pathological feature caused by the hyperphosphorylation of tau protein. Tau protein, transmitted by extracellular vesicles (EV) in the form of prions, accelerates the occurrence and development of AD (Noori et al., 2023). As described previously, neutral sphingomyelinase 2 (nSMase2) hydrolyzes sphingomyelinase to ceramides and serves as a key enzyme in the production of EV, thereby expediting the release and trafficking of tau protein (Tallon et al., 2021). Studies have shown that increased tau expression in PS19 and AAV-hTau transgenic mice, enhances nSMase2 activity and ceramide levels, promoting the formation of EV and the release and dissemination of tau protein, ultimately accelerating the damage of healthy neurons (Tallon et al., 2023). However, the deletion of nSMase2 in the familial AD transgenic mice model 5x FAD mice reduces ceramide levels and tau phosphorylation, ameliorating AD-related pathological changes (Tallon et al., 2023). Cambinol, a non-competitive nSMase2 inhibitor, hinders exosome-mediated tau protein transfer between cells and the spread of pathological forms of tau protein between cells by inhibiting nSMase2 activity, thereby slowing down the progression of AD (Zhu et al., 2021). PDDC, a highly selective, brain-permeable oral nSMase2 inhibitor, not only directly reduces tau propagation and tau phosphorylation, but also reduces hippocampal gliosis, neuronal and synaptic degeneration and normalizes brain ceramide levels (Tallon et al., 2023). Consequently, PDDC may be a potential novel strategy for the treatment of AD. However, the tolerability of PDDC requires further evaluation before advancing to clinical trials. In summary, ceramide and its metabolites exert an effect on tau protein and play an important role in the pathogenesis of AD.

### 4.3 Brain insulin resistance

The brain is one of the target organs for insulin, with insulin receptors distributed in most brain cells. Under normal conditions, insulin and IGF-1 inhibit glycogen synthesis kinase GSK3β by phosphorylating Akt to avoid excessive tau protein production through its phosphorylation (Hong and Lee, 1997). Insulin and IGF-1 also affect Aβ through a variety of ways. They inhibit the production of Aβ by suppressing the amyloid precursor protein cleaving enzyme BACE-1 and its substrate APP. Additionally, both insulin and IGF-1 prevent the accumulation of Aβ by enhancing the transport of Aβ binding carrier protein in the brain, and also prevent the accumulation of Aβ in the cell by accelerating the transport of Aβ from the Golgi to the plasma membrane (Carro et al., 2006; Yang and Song, 2013; Li et al., 2015; Kandimalla et al., 2017). Intraventricular injection of STZ has been demonstrated to induce insulin resistance in the brain and significantly reduce the insulin receptor IRS-2, accompanied by significant memory loss, Aβ deposition and tau phosphorylation. Therefore, brain insulin resistance can lead to Aβ deposition and tau phosphorylation, exacerbating the progression of AD (Abosharaf et al., 2024). The increase of ceramide in the CNS activates PP2A/PKCζ, inhibiting Akt/PKB signaling pathway. This impedes the translocation of GLUT4, a key molecule in the downstream pathway, to the plasma membrane, hindering effective glucose uptake in the brain and worsening brain insulin resistance (Grillo et al., 2009). In addition, ceramides also aggravate brain insulin resistance by activating the phosphorylation of MAPK and JNK, hindering insulin binding to the insulin receptor IRS-1 (Ma et al., 2009; Therease et al., 2012). Therefore, the increase of ceramide in the CNS aggravates brain insulin resistance, leading to Aβ deposition and tau phosphorylation, and plays an important role in the onset and development of AD.

The article "A review of the mechanisms of abnormal ceramide metabolism in type 2 diabetes mellitus, Alzheimer’s disease, and their co-morbidities" was published in 2024. Journal: Front Pharmacol.

### 4.4 Mitochondrial dysfunction

As previously mentioned, ceramides induce mitochondrial dysfunction, mainly in terms of abnormal energy metabolism, mitophagy, impaired kinetics, and transport defects. This mitochondrial dysfunction is also an important aspect in the pathogenesis of AD, which diminishes ATP production, disrupts neurotransmitter imbalance, amplifies ROS levels, hinders the removal of damaged mitochondria, thereby affecting synaptic activity and plasticity. This disruption damages synaptic function, hinders neurotransmission, and may even lead to neuronal apoptosis, contributing to the development of AD (Alshial et al., 2023).

Neurons, glial cells and synapses require substantial energy for effective neural signal transmission. Studies have shown that AD patients exhibit reduced activity and impaired dynamics of mitochondrial complexes in the brain, resulting in decreased ATP production and abnormal energy metabolism. This leads to weakened synaptic connections, reduced neurotransmission, and contribute to AD-related memory loss (Gowda et al., 2022). Ceramide has been shown to mediate insulin-induced mitochondrial bioenergetics damage in the brain of ApoE4 mice (Carr et al., 2023). In addition, mitochondrial dysfunction is also closely associated with oxidative stress and ROS that are neurotoxic during AD. Ceramide has been implicated in regulating oxidative phosphorylation and mitochondrial function, associated with decreased mitochondrial respiratory chain (MRC) activity, abnormal mitochondrial membrane potential, and increased ROS (Kogot-Levin and Saada, 2014). Oxidative stress may also result from the inhibition of mitochondrial respiration and ATP production by NADPH oxidase 4 (NOX4), which increases the damage of mitochondrial metabolism. Upregulation of NOX4 can promote mitochondrial ROS production, mitochondrial fragmentation and inhibit cellular antioxidant processes in human astrocytes to induce oxidative stress (Park et al., 2021). In addition, the ApoEε4 allele (ApoE4) is associated with many pathological processes in AD, such as Aβ and Tau abnormalities (Pires and Rego, 2023). Studies revealed that ApoE4 causes mitochondrial dysfunction and neurotoxicity, associated with increased mitochondrial Ca^2+^ and ROS levels (Mahley, 2023). Additionally, the increased brain mitochondrial membrane permeability in AD patients can release apoptosis-related proteins and activate the apoptosis signaling pathway (Gao et al., 2022). Accumulation of ceramide in the brains of AD patients is identified as a key mediator in the cascade of oxidative stress-driven neuronal apoptosis and Aβ-induced neuronal degeneration (Jazvinšćak Jembrek et al., 2015). In the context of aging or elevated blood glucose and lipid levels, mitochondrial dysfunction can damage antioxidant enzymes, increase ROS production, induce changes in mtDNA, and trigger oxidative stress, cell damage, and neuronal death (Misrani et al., 2021).

The article "A review of the mechanisms of abnormal ceramide metabolism in type 2 diabetes mellitus, Alzheimer’s disease, and their co-morbidities" was published in 2024. Journal: Front Pharmacol.

Taken together, ceramide-induced mitochondrial dysfunction contributes to multiple mechanisms in AD, encompassing decreased MRC activity, increased ROS production, oxidative stress, decreased mitochondrial membrane potential, ultimately leading to cell death and neurotransmission imbalance (Kogot-Levin and Saada, 2014).

### 4.5 Induction of neuroinflammation

Neuroinflammation constitutes a crucial mechanism in the progression of AD, with activated glial cells, including astrocytes and microglia, acting as both sources and targets of proinflammatory mediators (Heppner et al., 2015; de Wit et al., 2019). Elevated levels of sphingomyelin in the brain tissue of AD patients have been observed, and sphingomyelin hydrolysis by sphingomyelinase produces ceramides (Varma et al., 2018). The increased ceramide levels activate the NF-κB signal transduction in microglia, shifting the glial response towards inflammation and prompting the release of TNF-α, IL-1β, and IL-6 from astrocytes, thereby inducing neuroinflammation (de Wit et al., 2019). In microglia isolated from adult 5xFAD mice, inhibiting A-SMase has been found to reduce Aβ-induced release of proinflammatory cytokines like TNF-α, IL1-α, and C1q, which are implicated in inducing EV secretion by reactive astrocytes. Imipramine intervention in 5xFAD mice led to reduced pro-inflammatory microglia, reactive astrocytes, and neuronal death (Crivelli et al., 2023).

The article "A review of the mechanisms of abnormal ceramide metabolism in type 2 diabetes mellitus, Alzheimer’s disease, and their co-morbidities" was published in 2024. Journal: Front Pharmacol.

SPT is the first step in *de novo* ceramide synthesis, and blocking SPT activity also prevents astrocytes from synthesizing proinflammatory mediators such as IL-1β, TNF-α, iNOS, and COX-2 (De Vita et al., 2019). In addition, inhibition of SPT reduces the secretion of pro-inflammatory cytokines by astrocytes and inhibit the neurotoxicity of caspase-3 (De Vita et al., 2019). During chronic CNS inflammation, both ceramide and its derivative sphingolipid lactosylceramide increase in astrocytes, exacerbating inflammation and neurodegeneration (Mayo et al., 2014). Hence, abnormal ceramide metabolism in glial cells is intricately linked to the neuroinflammatory response, playing a pivotal role in the pathological mechanism of AD (Figure 3).

**FIGURE 3:** The pathogenesis of AD caused by ceramides.

## 5 Ceramide mediated the pathogenesis of T2DM combined with AD

In the preceding article, we discussed the role and mechanism of ceramides in the pathogenesis of T2DM and AD, respectively. However, as the global population ages, the co-occurrence of the two diseases is becoming a significant public health problem, necessitating an urgent investigation into the mechanisms governing their combination. T2DM is a risk factor for AD, and AD is one of the complications of T2DM. The dysfunction of cerebrovascular function in T2DM will seriously affect the clearance of brain’s metabolites by altering the integrity and elasticity of cerebral vessels. This process detrimentally damages the Aβ clearance system of blood vessels, leading to the deposition of Aβ in the brain (Ergul et al., 2012). These findings highlight a strong association between T2DM and AD. Insulin resistance, inflammation, amyloid accumulation, oxidative stress and mitochondrial dysfunction are common pathological features of T2DM and AD. Therefore, in recent years, some scholars have labeled AD as “type 3 diabetes” or “brain diabetes" (Nguyen et al., 2020; Michailidis et al., 2022; Fauzi et al., 2023a). However, the common factors and underlying molecular mechanisms driving these clinical phenomena remain unknown. Dysregulation of lipid metabolism leads to the accumulation of toxic lipids in the liver and visceral adipose tissue. With cell damage and death caused by ER stress and oxidative stress, toxic lipids are released into the circulation. Due to their lipid-soluble nature, they can cross the blood-brain barrier and cause neurotoxic damage, inflammation, insulin resistance, and neurodegeneration (de la Monte, 2012; de la Monte, 2009; Makki and Rahman, 2023). Studies have indicated that the abnormal metabolism of ceramide may lead to the disorder of various metabolic processes, serving as a crucial link in the common pathogenesis of T2DM and AD.

The article "A review of the mechanisms of abnormal ceramide metabolism in type 2 diabetes mellitus, Alzheimer’s disease, and their co-morbidities" was published in 2024. Journal: Front Pharmacol.

### 5.1 Insulin and IGF-1

Insulin is a glucose-regulating hormone present in both the peripheral and CNS, acting on the insulin receptor (InsR). The InsR plays an important role in regulating carbohydrate, lipid, protein metabolism, and controlling brain neurotransmitter levels (Verdile et al., 2015). In the normal brain, insulin signaling is essential for regulating glucose uptake and metabolism as a major energy source (Fauzi et al., 2023b). AD can be considered a central metabolic disease, partially due to impaired glucose metabolism. This impairment is associated with deficiencies in insulin and IGF signaling pathways in the brain, which are physiologically involved in energy production, neuronal survival, and plasticity and thus play a key role in cognition and memory (Blázquez et al., 2022). Persistent peripheral insulin resistance may lead to dysregulation of brain insulin receptor signaling. Studies have shown that both InsR and IGF-1R, along with their common downstream pathways, are widely distributed throughout the brain. They are regulators of brain function, whole-body energy balance, and metabolism (Kleinridders et al., 2014). Importantly, impairment in insulin signaling becomes evident years before the onset of AD and intensifies as the disease progresses (Steen et al., 2005). Consequently, studying insulin and insulin resistance becomes a crucial avenue for exploring the comorbidity of AD and T2DM(Sperling et al., 2011).

T2DM-related obesity induces hepatic insulin resistance, which lead to increased inflammation and metabolic dysfunction, resulting in dysregulated lipolysis and heightened ceramide production (Lyn-Cook et al., 2009). Elevated ceramide levels in turn promote ER stress in the liver, which aggravates insulin resistance, inflammation and oxidative stress (de la Monte, 2017). Studies have demonstrated a significant rise in ceramide levels in the liver, serum, and brain of mice and rats subjected to a prolonged high-fat diet, accompanied by the development of steatohepatitis and brain insulin resistance leading to neurodegeneration (Lyn-Cook et al., 2009; de la Monte et al., 2010). Cytotoxic ceramides generated in the periphery can traverse the blood-brain barrier (BBB) due to their hydrophobic and lipid-soluble nature. This leads to a substantial accumulation of ceramides in the central nervous system (CNS), exerting toxic effects. This accumulation results in reduced insulin signaling, increased proinflammatory cytokines, and the exacerbation of brain insulin resistance, neuronal apoptosis, and neuroinflammation (Saraya et al., 2023). In mice with high-fat diet induced T2DM, the mRNA expression of ceramides CER2, CER4, SPTLC1 and SPTLC2 increased in the liver, accompanied by mild neurodegeneration and brain insulin resistance. Notably, the high-fat diet did not elevate the expression of native ceramides in the brain. These findings suggest that brain insulin resistance in ceramide-mediated T2DM with AD may stem from peripheral insulin resistance (Lyn-Cook et al., 2009).

The article "A review of the mechanisms of abnormal ceramide metabolism in type 2 diabetes mellitus, Alzheimer’s disease, and their co-morbidities" was published in 2024. Journal: Front Pharmacol.

Ceramide activates PP2A, reducing the activity of Akt, damaging the insulin signaling pathway, and inducing peripheral insulin resistance. This is induced by the neurodegenerative liver brain axis and affects the CNS through the BBB, leading to cognitive impairment (de la Monte et al., 2010). PP2A is involved in both AD and T2DM, and its expression can be inhibited by insulin (Vogelsberg-Ragaglia et al., 2001; Clodfelder-Miller et al., 2006). Peripheral cytotoxic ceramides also contribute to neurodegeneration with impaired neuronal cell viability, energy metabolism, and insulin/IGF signaling (Tong and de la Monte, 2009). Intervention with synthetic C2Cer in rat pups led to hyperglycemia and hyperlipidemia, accompanied by increased serum ceramide levels. C2Cer could affect the expression and phosphorylation of insulin receptor, IGF-1 receptor, IRS-1 and Akt, leading to dysregulation of lipid metabolism and increased ceramide production. This disturbance further affected insulin and IGF signaling in the liver and brain. GAPDH, a key enzyme in the glycolytic pathway regulated by insulin, showed decreased expression, correlating with ceramide-mediated ATP damage. The observed effects resemble those induced by long-term high-fat diet feeding, including increased expression of insulin and IRS-4, decreased expression of CHAT and GAPDH, and heightened immunoreactivity of 4-HNE and ubiquitin (Moroz et al., 2008). It is evident that decreased GAPDH expression is associated with ceramide-mediated ATP damage (Alexander-Bridges et al., 1992). Ceramide also increased the expression of acetylcholinesterase (AChE) and AβPP-Aβ. Consequently, T2DM may establish a brain-centered cycle involving elevated levels of ceramide, TNF-α, and AβPP-Aβ, leading to progressive insulin resistance. This disruption in energy metabolism and acetylcholine homeostasis could further exacerbate AD (Tong and de la Monte, 2009).

### 5.2 Tau protein

As mentioned above, hyperphosphorylation of tau can cause neurofibrillary tangles (NFTS) leading to amyloid β plaques, an important histopathological feature of AD (Lacovich et al., 2017). Tau plays an important role in the peripheral nervous system and is implicated in the induction of insulin resistance and T2DM. Tau hyperphosphorylation has been identified in islets of T2DM and AD mice, emphasizing an additional link between T2DM and AD through abnormal tau protein metabolism (Bharadwaj et al., 2017).

The article "A review of the mechanisms of abnormal ceramide metabolism in type 2 diabetes mellitus, Alzheimer’s disease, and their co-morbidities" was published in 2024. Journal: Front Pharmacol.

Insulin and IGF-1 play a role in reducing tau phosphorylation in neurons by inhibiting GSK3 activity. GSK3, a constitutively active serine/threonine kinase with two isoforms (α and β), is widely expressed in tissues and involved in various cellular processes, including glycogen metabolism, gene transcription, apoptosis, neuronal function, and microtubule stability (Bhat et al., 2003). GSK3 phosphorylates a large number of substrates, particularly tau, a neuronal protein directly associated with AD (Bhat et al., 2003; Schubert et al., 2004; de la Monte et al., 2011). Impaired insulin and IGF signaling may result in the overactivity of certain kinases and phosphatases, leading to decreased tau expression and hyperphosphorylation, GSK-3β, a kinase known to phosphorylate tau, is particularly significant in this context. It has also been demonstrated that mice on a high-fat diet exhibited inhibited GSK3 activation through the Akt/PKB pathway after blocking of the *de novo* ceramide synthesis and rescue pathway, thereby limiting their ability to phosphorylate tau and reducing Aβ deposition (Charytoniuk et al., 2021). Apart from hyperphosphorylation, impaired insulin and IGF signaling also alters expression encoded by tau genes. These abnormalities ultimately lead to synaptic and mitochondrial dysfunction and progressive neurodegeneration in AD (Hong and Lee, 1997). It has been observed that reducing ceramide accumulation can alleviate brain insulin resistance and tau protein phosphorylation, offering potential benefits for AD recovery.

### 5.3 Neuroinflammation

There exists a close interaction between ceramides and various inflammatory factors (Li, 2022). In T2DM, insulin resistance is closely associated with elevated levels of inflammatory mediators. Elevated levels of inflammatory markers result in a dysfunctional immune response, subsequently inducing insulin resistance. Numerous studies have suggested that neuroinflammation is a primary contributor to insulin resistance in the brain of AD patients (Bosco et al., 2011). Consistent with this, the activation of inflammatory markers can be detected prior to the manifestation of clinical symptoms in AD and is involved in the lesion development. The accumulation of inflammatory mediators is also observable in AD patients. In chronic neuroinflammation, microglia are activated after engulfing Aβ, releasing IL-1β, IL-6 and TNF-α concurrently. These inflammatory factors accelerate the pathological process of neuron loss in AD patients (Rosenberg, 2005). However, studies conducted on primary rat astrocytes showed that ceramide could stimulate the expression of pro-inflammatory molecules such as TNF-α and the activation of NF-κB (Gu et al., 2013). Moreover, peripheral insulin resistance induced by T2DM and obesity also generates high levels of cytotoxic lipids, including ceramides, which traverse the BBB and contribute to insulin resistance and neuroinflammation in the brain (de la Monte, 2009). Simultaneously, research has established a close relationship between peripheral inflammation and CNS inflammation, which is a key factor driving the progression of T2DM and AD (Estato et al., 2013; Kacířová et al., 2020; Khan and Hegde, 2020). Proinflammatory cytokines are highly activated in T2DM and AD, and this mechanism stimulates ceramide synthesis, allowing it to play a pivotal role in both T2DM and CNS diseases.

The article "A review of the mechanisms of abnormal ceramide metabolism in type 2 diabetes mellitus, Alzheimer’s disease, and their co-morbidities" was published in 2024. Journal: Front Pharmacol.

The activation of microglia induced by Aβ can trigger the release of various inflammatory cytokines, which is one of the important processes involved in neuroinflammation (Rosenberg, 2005). Neuroinflammation is implicated in the deterioration of synaptic function, inhibition of hippocampal neurogenesis, acceleration of neuronal death, and induction of Aβ and inflammatory mediators through the BBB(Sekeljic et al., 2012). Furthermore, it recruits white blood cells to the CNS, fostering neurodegeneration and initiating a detrimental cycle of chronic inflammation. This cycle mediates the intricate relationship between T2DM and AD. Animal studies have found that liver steatosis in HFD mice is accompanied by patchy lymphocytic nuclear cell inflammation. Additionally, the level of ceramide in the liver of HFD mice is significantly higher than that in LFD mice. The proinflammatory cytokine TNF-α increased in the serum of HFD mice, while the temporal cortex and hippocampus of HFD mice showed sustained neuronal shrinkage, apoptosis and decreased cell density. These findings indicates that ceramide levels increased in the presence of insulin resistance, promoting oxidative stress. This, in turn, triggers the activation of the proinflammatory cascade in astrocytes, impacting the CNS(Lyn-Cook et al., 2009).

NLRP3 is a multimer protein complex that induces pyroptosis and trigger the release of proinflammatory cytokine IL-1β, which not only promotes the deposition of Aβ, but also leads to the hyperphosphorylation of tau protein (Naeem et al., 2023). NLRP3 inflammasome can be regulated by ceramide, which activates caspase-1 in macrophages and adipose tissue, stimulates the release of IL-1β and IL-18, and leads to pyroptosis and endothelial cell death (Lee et al., 2016; Liu F. et al., 2022; Pizzuto et al., 2022). Therefore, an increase in ceramide levels disrupts vascular endothelial function and increases vascular permeability (Liu F. et al., 2022). Transcriptomic studies have uncovered neuroinflammation, endothelial dysfunction, and changes in vascular permeability in the brains of T2DM mice (Nuthikattu et al., 2024). In T2DM patients, the NLRP3 inflammasome is significantly higher than in normal individuals, posing a risk for secondary cognitive impairment. The primary mechanism is believed to be T2DM-mediated neuroinflammation, which increases the permeability of BBB(Tian et al., 2022). In a mouse model of AD, inhibition of NLRP3 inflammasome activity not only reduced Aβ content, but also reduced proinflammatory cytokine production as well as mitigating cognitive impairment (Li et al., 2024). Therefore, the increase of ceramide is an inducing factor for insulin resistance and various inflammatory factors, which will lead to the T2DM aggravation, exacerbating neuroinflammation, damage neurons and worsening AD.

The article "A review of the mechanisms of abnormal ceramide metabolism in type 2 diabetes mellitus, Alzheimer’s disease, and their co-morbidities" was published in 2024. Journal: Front Pharmacol.

### 5.4 Oxidative stress and mitochondrial dysfunction

BBB functions as a dynamic barrier regulating substance exchange between the peripheral and central nervous system (CNS), crucial for maintaining brain homeostasis and protection (Mora et al., 2020). Following BBB injury, peripheral oxidative stress induced by hyperglycemia can trigger the release of excessive ROS from neuronal mitochondria, leading to neuronal apoptosis. Oxidative stress results from an imbalance between ROS, reactive nitrogen free radicals (RNS), antioxidants, and pro-oxidants, causing disruptions in REDOX pathways and metabolic processes. Prolonged oxidative stress exacerbates tissue and organ oxidative damage (Di Meo et al., 2016; Pizzino et al., 2017). Oxidative stress can affect the antioxidant capacity of cells, leading to the peroxidation of proteins, lipids and mitochondria, contributing to T2DM and AD (Valko et al., 2007). Increased derivatives of oxidative stress have been observed in plasma, fat, liver, skeletal muscle, and brain tissue during insulin resistance (Maciejczyk et al., 2018). The human brain, with its high lipid content, elevated oxygen consumption rate, and low antioxidant capacity, is particularly vulnerable to oxidative stress (Butterfield et al., 2006). AD-related membrane lipid metabolism disorders partly result from increased Aβ production or deposition (Cutler et al., 2004). Elevated ceramide levels, triggered by Aβ-induced oxidative stress, contribute to hippocampal neuron death. Additionally, abnormal glucose metabolism in the liver increases ROS and RNS production, inflammatory cytokines, and impacts the CNS(Mahboobi et al., 2014).

The article "A review of the mechanisms of abnormal ceramide metabolism in type 2 diabetes mellitus, Alzheimer’s disease, and their co-morbidities" was published in 2024. Journal: Front Pharmacol.

Chronic hyperglycemia-induced elevated mitochondrial fission can exacerbate mitochondrial morphology and dysfunction, ultimately impairing neuronal synaptic plasticity in T2DM(Edwards et al., 2010). The imbalance of mitochondrial homeostasis further contributes to synaptic damage and cognitive deficits in diabetic patients (Zhou et al., 2018). Resveratrol has demonstrated its efficacy to prevent mitochondrial dysfunction and protect against diabetes-induced cognitive dysfunction (Cao et al., 2023). Moreover, the increase in ceramide levels significantly inhibits mitophagy regulated by PINK1/Parkin pathway, further hindering the efficient removal of damaged mitochondria, resulting in aggravated mitochondrial dysfunction and metabolic disorders (Wang X. et al., 2023) (Figure 4).

**FIGURE 4:** Ceramide mediated the pathogenesis of T2DM combined with AD.

## 6 Regulatory ceramide can be used as a therapeutic target for T2DM combined with AD

Based on the above, ceramides have a common important role in the pathogenesis of T2DM and AD, so it is of strong clinical practical significance to study ceramides as a diagnostic and therapeutic target for both diseases. In this context, the regulation of ceramide involves two main pathways: inhibiting ceramide synthesis and reducing ceramide deposition.

Previous studies have identified a range of ceramide synthase inhibitors with the ability to selectively target distinct CerS isoforms. Fumonisins B1 is one of the first CerS inhibitors derived from the fusarium toxin family and implicated in the pathogenesis of human esophageal cancer (Régnier et al., 2019). However, fumonisin B1 has a certain degree of hepatotoxicity, which limits its clinical application (Dellafiora et al., 2018). In addition, Turner et al. discovered that P053, a selective CerS inhibitor that specifically inhibits CerS1 expression, exhibits the potential to ameliorate insulin resistance by diminishing C18:0 ceramide levels in both cells and skeletal muscle of mice (Turner et al., 2018). Cannabigerol, one of the cannabinoid compounds contained in the cannabis leaf, is a psychotropic drug. Cannabinoid can increase the phosphorylation of Akt at Thr34 by inhibiting the *de novo* synthesis of ceramide, increase the activity of Akt enzyme and inactivate GSK-3β enzyme, thereby improving hepatic insulin sensitivity and treating insulin resistance in obese animal models (Bzdęga et al., 2023). Cannabinoid has shown the potential to reduce tau protein phosphorylation and ameliorate Aβ deposition. Furthermore, CB1R inhibitor, while suppressing SPT activity, CerS1, and CerS6 expression, effectively reduces hepatic ceramide content (Cinar et al., 2014). However, due to its brain permeability and associated psychiatric side effects, it remains unused in clinical practice.

The article "A review of the mechanisms of abnormal ceramide metabolism in type 2 diabetes mellitus, Alzheimer’s disease, and their co-morbidities" was published in 2024. Journal: Front Pharmacol.

SPT, a pivotal enzyme in ceramide synthesis, represents the initial stage in the biosynthesis of diverse sphingolipids, and inhibiting SPT can curtail ceramide production. Myristoin is a widely studied SPT inhibitor that irreversibly inhibits SPT expression and reduces ceramide levels. In skeletal muscle of mice, myristoin-mediated SPT inhibition restored protein homeostasis and mitochondrial function (Lima et al., 2023). Bisphenol A (BPA) has been shown to be an important contributor to insulin resistance and metabolic diseases. Myristoin has been demonstrated to inhibit BPA-induced ceramide increase, consequently reducing inflammatory factors IL-1β and TNF-α(Zabielski et al., 2019; Wang G. et al., 2023). Human skeletal myoblast studies revealed that myristoin treatment inhibited palmitic acid-induced glycogen synthesis and was found to be associated with a significant reduction in ceramide content, while intracellular DAG levels remained elevated (Pickersgill et al., 2007). L-cycloserine, another SPT inhibitor. Exhibited the ability to reduce fasting blood glucose and plasma insulin levels, enhance Akt phosphorylation in the soleus muscle of JCR obese rats, and improve insulin signaling (Fillmore et al., 2015). Treatment with myristicin and l-cycloserine in L6 myotubes prevented palmitate-mediated increase in intracellular ceramide content, increased Akt phosphorylation at Thr34, and attenuated palmitate-induced insulin resistance (Powell et al., 2004). Diabetic nephropathy is characterized by podocyte injury, and myristoin has been shown to diminish mitochondrial ceramide accumulation in podocytes, thereby alleviating podocyte injury (Woo et al., 2020).

Myristoin is abundant in many fungi, such as Cordyceps sinensis. Cordyceps sinensis, a traditional Chinese medicine, has the functions of lowering blood glucose, anti-inflammation, anti-oxidation, regulating immune function, and regulating cell apoptosis (Liu W. et al., 2022). It has a significant adjuvant treatment effect on chronic progressive diseases such as T2DM. Recent animal experiments have shown that Cordyceps sinensis extract containing myristicin significantly reduced serum ceramide content, alleviated liver steatosis, increased insulin sensitivity and improved insulin sensitivity in obese mice. In addition, Cordyceps sinensis extract did not induce intestinal toxicity or alter intestinal morphology during the intervention, common side effects of conventional SPT inhibitors (Li et al., 2022). This suggested that Cordyceps sinensis extract containing myristoin can inhibit ceramide synthesis, making edible Cordyceps sinensis a potential supplement for treating metabolic diseases. However, controlled clinical studies are necessary in the future to ascertain the safety and efficacy of cordyceps treatment as a ceramide inhibitor for metabolic improvement.

The article "A review of the mechanisms of abnormal ceramide metabolism in type 2 diabetes mellitus, Alzheimer’s disease, and their co-morbidities" was published in 2024. Journal: Front Pharmacol.

There is limited research on reducing ceramide deposition. It is understood that excessive FFA deposition in the body can stimulate the synthesis of ceramide in cells and tissues. Inhibiting FFA release may emerge as a strategy to modulate ceramide and decelerate the progression of metabolism-related diseases. Fenofibrate, a commonly used lipid-regulating drug primarily employed in treating hyperlipidemia, has not traditionally been utilized for T2DM and AD treatment. Recent studies revealed that fenofibrate slowed the development of chronic inflammation by inhibiting hepatic ceramide synthase and reducing the accumulation of ceramide and lipids in plasma and liver (Camacho-Muñoz et al., 2021). Saroglitazar and heparin, typically prescribed for hyperlipidemia, have exhibited promising inhibitory effects on ceramides in recent studies (Sarkar et al., 2021). Consequently, these drugs hold potential for reducing ceramide deposition and may become candidates for treating the comorbidity of the two diseases. However, further clinical research is essential to confirm these findings.

The regulation of ceramide has found practical application in clinical treatment, particularly in managing skin diseases. The outermost layer of the skin is the stratum corneum, and ceramides, as part of lipids, are an important component of the stratum corneum and play a protective role in skin barrier function (Menon et al., 2012). Products such as cleansers and moisturizers containing ceramides, commonly used as an adjunct to the treatment of skin conditions such as acne, improve the skin barrier function and reduce skin irritation (Bouwstra et al., 2023; Gold et al., 2024). Therefore, if the long-term use of ceramide inhibitors may lead to side effects such as skin barrier damage, ceramide as a therapeutic target has some complexity, which needs to be further explored by researchers in the future.

## 7 Conclusion and the future direction

The biological effects of sphingolipids are diverse and involved in various diseases, including inflammation, autoimmune diseases, tumors, diabetes, and insulin resistance.

Ceramide, positioned at the center of sphingolipid metabolism, acts as a second messenger in cells and participates in a variety of signal transduction that affect the disease process. Numerous enzymes involved in ceramide synthesis or metabolism have emerged as potential therapeutic targets for metabolic diseases. Ceramide’s pivotal role in the comorbidity of T2DM and AD is evident; it regulates classical insulin signaling pathways like the PP2A/AKT pathway, directly or indirectly impacting disease progression. Consequently, elucidating the mechanisms underlying the comorbidity of these two diseases and regulating their metabolic processes holds promise for future treatments. Targeted ceramide inhibitors have demonstrated significant efficacy in animal experimental studies, potentially evolving into future drugs for treating the comorbidity of T2DM and AD. However, bridging the gap to meet clinical practice requirements remains a considerable challenge.

The article "A review of the mechanisms of abnormal ceramide metabolism in type 2 diabetes mellitus, Alzheimer’s disease, and their co-morbidities" was published in 2024. Journal: Front Pharmacol.

At present, basic research on multimorbidity has not made a breakthrough, with mainstream research predominantly centered around single disease models. Modeling methods and intervention evaluation for multimorbidity models lack reported, and multiple key link mechanisms remain to be clarified. In the short term, exploring new effects of mature drugs widely used in clinical practice may prove a more reliable approach. For instance, metformin, as a first-line treatment for T2DM, has demonstrated positive on improving cognitive impairment in mice models induced by inflammatory factors (Zhu et al., 2023). However, this evidence is animal-model-based, and it remains uncertain whether the effect is related to ceramide regulation. In summary, the identified challenges necessitate further clinical research to furnish sufficient evidence, posing a significant challenge for precise treatment of comorbidities based on ceramide regulation in the future. Researchers in related fields need to persist in their exploration of these complexities.
